This article has been retracted.

# Design and Application of Electronic Rehabilitation Medical Record (ERMR) Sharing Scheme Based on Blockchain Technology

**DOI:** 10.1155/2021/3540830

**Published:** 2021-08-27

**Authors:** Jing Zhang, Zhenjing Li, Rong Tan, Cong Liu

**Affiliations:** ^1^Faculty of Business Information, Shanghai Business School, 201400, China; ^2^Rehabilitation Department, Hannover Medical School, 30625, Germany; ^3^Rehabilitation Department, Shenzhen Longhua District Central Hospital, 518110, China

## Abstract

As the value of blockchain has been widely recognized, more and more industries are proposing their blockchain solutions, including the rehabilitation medical industry. Blockchain can play a powerful role in the field of rehabilitation medicine, bringing a new research idea to the management of rehabilitation medical data. The electronic rehabilitation medical record (ERMR) contains rich data dimensions, which can provide comprehensive and accurate information for assessing the health of patients, thereby enhancing the effect of rehabilitation treatment. This paper analyzed the data characteristics of ERMR and the application requirements of blockchain in rehabilitation medicine. Based on the basic principles of blockchain, the technical advantages of blockchain used in ERMR sharing have been studied. In addition, this paper designed a blockchain-based ERMR sharing scheme in detail, using the specific technologies of blockchain such as hybrid P2P network, block-chain data structure, asymmetric encryption algorithm, digital signature, and Raft consensus algorithm to achieve distributed storage, data security, privacy protection, data consistency, data traceability, and data ownership in the process of ERMR sharing. The research results of this paper have important practical significance for realizing the safe and efficient sharing of ERMR, and can provide important technical references for the management of rehabilitation medical data with broad application prospects

## 1. Introduction

With the rapid development of the rehabilitation medical industry and the rapid increase of rehabilitation medical data, many medical institutions have begun to use electronic rehabilitation medical record (ERMR) to record the status of patients receiving rehabilitation services. Rehabilitation medical record comprehensively records the patient's identity information, medical history, examination results, and the evaluation, diagnosis, and training of rehabilitation medicine. It is an important part of rehabilitation medical work and determines the overall quality of rehabilitation medical treatment. ERMR can provide more convenient storage and query for rehabilitation medical data and store more comprehensive diagnosis information. At the time of diagnosis, the rehabilitation doctor can quickly and accurately understand the patient's medical history through the ERMR, so as to make a more comprehensive and accurate analysis and assessment of the patient's condition.

For comprehensive complex diseases, chronic diseases, and dysfunctions (such as stroke, spinal cord injury, fractures, and osteoarthropathy), patients often need long-term, continuous diagnosis and treatment. A safe, reliable, and easily accessible ERMR will definitely improve the work efficiency of rehabilitation doctors, facilitate the rehabilitation doctors to accurately understand the patient's personalized information and rehabilitation needs, adopt targeted rehabilitation treatment plans, and improve the effectiveness of individual rehabilitation [1]. The sharing of ERMR is also beneficial to rehabilitation research institutions and provides basic data and case references for prospective scientific research [2, 3].

Blockchain is a new distributed infrastructure and computing model which uses the block-chain data structure to verify and store data, uses the distributed nodes and the consensus algorithms to generate and update data, uses the cryptography to ensure the security of data transmission and access, and uses the smart contracts composed of automated script codes to program and manipulate data. As a new computing model that builds trust at a low cost in an untrusted competitive environment, blockchain technology is considered a subversive innovation of computing model. It is changing the application scenarios and operating rules of many industries and is triggering a new technological innovation and industrial transformation on a global scale.

Blockchain is originated from encrypted digital currency and is currently being extended to other fields. As the value of blockchain is widely recognized, more and more industries are proposing their own blockchain solutions, including the medical and health industry. Blockchain can play a very powerful role in the medical field, which is particularly obvious in medical data management [4]. Blockchain is essentially a decentralized distributed storage system, which has great advantages in trust mechanism, data security, privacy protection, etc. Applying it to ERMR sharing will be a good breakthrough point with broad application prospects [5–7].

The application of blockchain technology to the processing of electronic medical data is one of the current hot areas of blockchain research. Electronic medical records can be stored in the blockchain system. However, if all medical data is directly stored in the blockchain network, it will increase the burden of calculation and storage on the blockchain. In order to solve these problems, many related research and applications have adopted a hybrid storage architecture, storing the original medical data in a local database, and only the index of the original data (i.e., the location of the local database) is stored on the blockchain. Zhang and Lin proposed a blockchain-based secure and privacy-preserving personal health information (PHI) sharing scheme for diagnosis improvements in e-Health systems and constructed two kinds of blockchains (namely the private blockchain and the consortium blockchain) by devising their data structures and consensus mechanisms [8]. Shamshad et al. put forward a blockchain-based privacy and security preserving electronic health record (EHR) sharing protocol and constructed two types of blockchains, in which the private blockchain was in charge of storing the EHRs, while the consortium blockchain storing the EHRs' secure indexes [9].

ERMR contains the patient's personal information; so, the confidentiality and security of the data should be ensured when the blockchain technology is applied to electronic medical record sharing. The encryption technology of the blockchain can be used to securely share data between authorized users. Dagher et al. proposed a blockchain-based framework for secure, interoperable and efficient access to medical records by patients, providers, and third parties, while preserving the privacy of patients' sensitive information. The framework utilized smart contracts in an Ethereum-based blockchain for heightened access control and obfuscation of data and employed advanced cryptographic techniques for further security [10]. Haque et al. used the SHA256 secure hash algorithm for generating a unique and identical 256-bit or 32-byte hash value for a particular medical record and focused on five mechanisms (i.e., digital access rules, data aggregation, data immutability, data liquidity, and patient identity) of data transition for securing the medical records at the proposed blockchain model [11].

In the blockchain network, since there is no trusted central authority, reaching a consensus between untrusted nodes is an important issue. Sri and Bhaskari proposed a blockchain-based encryption of patient data among shared network and used the consensus mechanism to validate Proof of Word and interoperability for data discovery and access [12]. Huang et al. proposed a blockchain-based privacy-preserving scheme which realized the secure sharing of medical data and executed a distributed consensus based on PBFT algorithm for transactions between patients and research institutions according to the prearranged terms [13]. Qazi et al. proposed a consensus algorithm titled Proof of Authenticity over the distributed platform for all medical stakeholders, in which hospitals and clinics are assumed the roles of both miners and validators, and designed a smart contract that follows the proof of authenticity mechanism [14].

The Hyperledger Fabric open-source project implements an underlying general framework of the permissioned blockchain, providing scalable applications such as identity verification, P2P protocol, access control, consensus algorithm, and smart contract and can support the application scenarios of blockchain in electronic medical record sharing. CLIM et al. proposed that the access control in the mobile health application can be implemented by using a permissioned blockchain built on the Hyperledger Fabric [15]. Sharma and Balamurugan used a blockchain-based framework Hyperledger Fabric and Composer tool to implement a blockchain-based electronic health record (EHR) network which made the EHRs more secure and private [16]. Usman and Qamar implemented a prototype of Electronic Medical Record Management System using permissioned blockchain platform “Hyperledger” which ensured the security, privacy, and easy accessibility of data [17].

The number of relevant literatures on the application of blockchain technology to the management of electronic medical records has shown a surge, but as far as its research content is concerned, it still has obvious limitations. The vast majority of the existing literatures are technical papers, focusing on the details of blockchain technology, but lack of discussion on the concept, connotation, and management method evolution of electronic medical record in the new technical environment. The existing literature often selects a single technical problem for detailed research, such as the privacy protection of electronic medical record,or the improvement of consensus algorithms, but it lacks the overall and systematic design of blockchain solutions and integrated research framework. The implementation of blockchain solutions in the existing literature mostly stays at the stage of simulation experiments, lacking practical considerations for specific application scenarios. Research on typical industry application cases is rarely involved, and there is a lack of exploratory thinking about the policy and laws that may be faced by the application of the solution. The application of blockchain in the management of electronic medical record is not only a technical issue, but more importantly, it is to study how blockchain creates value in practical applications and how to play its role in reducing costs, improving efficiency, and optimizing the integrity environment.

Based on the application requirements of data sharing in the field of rehabilitation medicine, the data characteristics of ERMR, and the basic principles of blockchain technology, this paper analyzed the technical advantages of blockchain used in ERMR sharing and designed a set of ERMR sharing scheme based on blockchain technology in detail to truly realize the distributed secure storage and sharing of rehabilitation medical data. Comparing the scheme in this paper with some existing blockchain-based medical data sharing schemes, this scheme has greater advantages in data security, system controllability, processing efficiency, etc. This paper deeply integrated blockchain technology and ERMR management, which helped solve the practical problems faced by ERMR management, realized the safe sharing of ERMR, and reduced the cost of ERMR collection, thereby facilitating the technology and efficiency transformation of health care industry and promoting the overall development of the health care service system. In addition, on the basis of theoretical research, this paper made full use of advanced computer technology to design and develop the overall scheme and typical application scenario of the ERMR management based on the blockchain, which will help guide the specific application of blockchain in the health and medical industry, and provide a technical path with industry reference value.

## 2. Application Requirements of Blockchain in ERMR Sharing

### 2.1. The Characteristics of Rehabilitation Medical Data

Rehabilitation medicine focuses on the overall rehabilitation of dysfunction, involving the comprehensive and coordinated application of multiple rehabilitation treatments such as physical therapy, occupational therapy, psychotherapy, drug therapy, and plastic therapy. It is usually a long-term treatment. Therefore, the data dimensions of ERMR are more abundant than ordinary clinical medical record, and provide comprehensive and accurate information for the overall assessment of the patient's health status.

Through literature review [18–20], as well as the collection and analysis of the hospitals' rehabilitation medical records, the main data content of the rehabilitation medical records can be summarized as shown in Table 1.

### 2.2. The Main Problems in ERMR Sharing

ERMR can comprehensively reflect the patient's functional level, health status, living status, etc. It not only involves rehabilitation medical institutions but also involves some important civil affairs departments and social functions [21, 22], such as social welfare, community services, social security for people with disabilities, education, employment, and charities aid. However, from the current situation, ERMR has not yet achieved safe and efficient sharing between different institutions. The main reasons are as follows.

Trust issues. In order to maintain the security of ERMR, doctors and patients will be strictly restricted when accessing data, and a lot of time and resources are needed to conduct permission review and verification. ERMR is a valuable data asset of rehabilitation medical institutions, and external sharing may reduce their own competitive advantages. There is a lack of a reasonable mutual trust mechanism between the owners and users of rehabilitation medical data. The lack of trust has caused serious isolated islands of medical information and hindered the development of medical big data and smart healthcare.

Security of rehabilitation medical data. In the traditional way, ERMR is usually stored in the local database of hospitals. In this centralized storage method, the amount of information in the local database of each hospital is huge [23], which is easy to become a key target of hacker attacks, leading to data leakage and data tampering.

The ownership of rehabilitation medical data. ERMR records the patient's vital data [24]. In theory, the patient should enjoy the priority data ownership. However, the current actual situation is that ERMR is controlled by medical institutions, and patients do not have the actual control capabilities of processing, using, and sharing their own ERMR. Obviously, this mechanism does not reasonably protect the rights and interests of information subjects.

The contradiction between ERMR sharing and patient privacy protection. With the rapid development of the Internet and big data technology, personal information protection has become a focus of attention worldwide. ERMR contains a large amount of sensitive and confidential personal information. Once leaked, it will cause serious data security risks and conflicts between doctors and patients. When ERMR is shared, privacy protection must be strengthened to prevent the leakage of patients' personal information.

The quality of rehabilitation medical data. Since ERMR involves the patient's vital data, the correctness, completeness, and real-time of the data are crucial to the patient's diagnosis and treatment effect. Once the wrong data or false data is entered, it will have a serious negative impact on diagnosis and treatment. Therefore, it is of great significance to implement strict medical data quality management and data traceability. However, because the technical standards of various rehabilitation medical institutions are not uniform, it is difficult to ensure the consistency of rehabilitation medical data, which increases the difficulty of medical information sharing.

With the rise of cloud computing technology, medical institutions can upload ERMR to a third-party cloud server, and the ERMR can be hosted by a third-party cloud service agency [25]. This method improves the efficiency of storage, retrieval, and sharing of ERMR to a certain extent. However, cloud servers are generally considered semitrusted. When all the rehabilitation medical data are stored in a centralized cloud server, once the cloud server is not well supervised or suffers a targeted malicious attack, it will cause all the rehabilitation medical data to be leaked, tampered, or even lost. The consequences will be very serious.

### 2.3. The Advantages of Applying Blockchain to ERMR Sharing

The P2P (peer-to-peer) network structure of blockchain can realize the distributed storage of ERMR. Distributed storage of massive ERMRs on multiple servers can effectively use the large and scattered storage and computing resources in the network, achieving the mass storage and high-performance computing of rehabilitation medical data [26]. There is no centralized node in the P2P network. Even if one of the nodes fails, it will not affect the normal operation of the entire blockchain system;so, the stability of the system is superior. Nodes can directly transmit data without going through a third-party centralized node, which can effectively reduce the risk of information leakage.

The blockchain data structure of the blockchain can ensure that the ERMR cannot be tampered with and can be traced. Under the blockchain data structure, blocks are created in chronological order and are connected into a chain by hash value, which can be traced back to the first block. The blockchain data structure can ensure that the ERMR cannot be tampered with, so that the original rehabilitation medical data maintains a high degree of consistency and integrity [27]. The timestamp in the block records the generation time of each block and the entry time of each medical data, making it easier to trace medical data and further increasing the difficulty of tampering with data, providing more credible and comprehensive protection for the ERMR.

The hash function of the blockchain can realize the privacy protection of patients. The hash encryption function can map the rehabilitation medical data into a string of garbled hash values composed of numbers and letters, and there is no way to reverse and decrypt it. The hash function can be used to encrypt personal identification data and sensitive data in the ERMR and strengthen the privacy protection of patients.

The asymmetric encryption algorithm and digital signature of the blockchain can strengthen the security of rehabilitation medical data. The asymmetric encryption algorithm uses public and private keys to encrypt and decrypt data, respectively, greatly reducing the risk of information leakage during information transmission, thereby ensuring the security of ERMR. Digital signature technology can realize user identity verification and prevent unauthorized users from accessing the ERMR.

The consensus mechanism of the blockchain can achieve “trust-free” and better promote the participation of medical institutions in ERMR sharing. The consensus mechanism solves the trust problem through mathematical algorithms and forms a new type of trust mechanism without the mutual trust between medical institutions [28]. At the same time, medical data ownership issues can be determined through the consensus mechanism, making medical data truly an asset with clear property rights and clear value.

## 3. Basic Principles of Blockchain Technology

Blockchain is not a single information technology, but an innovative combination of existing information technologies such as distributed data storage, point-to-point transmission, consensus mechanism, and encryption algorithm, so as to realize a new application mode in the Internet era. It has the technical characteristics of distributed storage, partial decentralization, quasianonymity, security, credibility, open source, and programmability, which can solve the difficult problems in the ERMR sharing in a targeted manner.

### 3.1. Peer-to-Peer (P2P) Network

The blockchain uses a peer-to-peer (P2P) network structure (see Figure 1) to organize all network nodes. It does not have a centralized node, but uses distributed storage technology, and each node stores a copy of the complete data. It can be seen that the blockchain is essentially a decentralized distributed database, and the block data is stored by all nodes in the blockchain system.

### 3.2. The Blockchain Data Structure

In the blockchain, data is organized and stored in a blockchain data structure. Each block can be divided into two parts, the block header and the block body. The blocks are created in chronological order and connected into a chain by block hash (also called block ID), as shown in Figure 2. The block header records the control information such as block version, block height, block hash, previous block hash, Merkle tree root, block timestamp, difficulty, and block nonce. The block body contains all the specific transaction data in this block and is stored in a Merkle tree structure. The leaf nodes are paired in pairs, and the hash operation is performed upwards until the root of the Merkle tree in the block header.

### 3.3. The Hash Encryption Function

The hash algorithm is one of the core technologies of blockchain. It is a collective name for a series of hash encryption functions. Through the hash function, the transaction information of any length in the block can be mapped into a series of fixed length hash values (similar to garbled codes) composed of numbers and letters, thereby hiding specific information. For example, the SHA-256 algorithm can convert the transaction data of any length into a string of 64 numbers or letters. The hash function is one-way and cannot be reversed and decrypted. It can be used to encrypt identity data and sensitive data to strengthen the privacy protection of the information subject.

The transaction data in the block body is hashed upward in a pairwise manner in the Merkle tree. This storage method can ensure that the transaction data cannot be tampered with. Once a piece of transaction data is modified, the Merkle tree of the block needs to be hashed again, so that the Merkle tree root and the block hash in the block header are changed and no longer match the next block.

### 3.4. The Asymmetric Encryption Algorithm

Each node in the blockchain has a unique pair of public and private keys. The public key is open to the outside world, indicating the identity of the node, and the private key is not open, indicating the right to control the information. Information encrypted with one of the keys can only be decrypted by the corresponding other key. The basic principle of asymmetric encryption algorithm is shown in Figure 3. When sending information, the sender A uses the public key of the receiver B to encrypt the information, and the information is transmitted on the network in the form of ciphertext. After receiving the information, the receiver B uses its private key to decrypt the information.

### 3.5. The Consensus Mechanism

The consensus mechanism is a mechanism that uses mathematical algorithms to create trust between nodes without central control. The data in the blockchain system is stored independently by all nodes. Under the coordination of the consensus mechanism, the data consistency of each node can be guaranteed. The consensus algorithm of the public blockchain is represented by Proof of Work (PoW), Proof of Stake (PoS), and Delegated Proof of Stake (DPoS), and the data writing order adopts the “write first and then consensus” method. The consensus algorithms of the private blockchain and the consortium blockchain mainly include Practical Byzantine Fault Tolerance (PBFT) and Raft, using the “consensus first and then write” data writing sequence.

### 3.6. The Smart Contract

Smart contract is the computer program deployed on the blockchain. It implements, compiles, and deploys the business logic of the blockchain system in the form of program code. Once the established conditions are met, it can be triggered and automatically executed, minimizing the manual intervention. The smart contracts of mainstream blockchain platforms are shown in Table 2.

## 4. Materials and Methods

### 4.1. The Network Structure Design

In order to realize the safe sharing of rehabilitation medical data under the premise of ensuring system controllability, in terms of network structure, a “partially decentralized” hybrid P2P network model can be adopted, as shown in Figure 4. Rehabilitation hospitals, rehabilitation centers, rehabilitation research institutes, insurance companies, regulatory authorities, and other institutions act as super nodes in a distributed network to form a consortium blockchain. Each super node and several ordinary nodes (i.e., patients) form a partial centralized network centered on the medical institution. Hybrid P2P network has a flexible structure and is less difficult to implement, which is more common in practical applications.

### 4.2. The Data Storage Design

In a hybrid P2P network, in order to ensure the security of the data on the blockchain and overcome the storage space limitations and performance bottlenecks of the blockchain, an on-chain-off-chain hybrid storage mechanism can be used. The ERMR can be divided into two parts: the detailed information and the summary information. The detailed ERMR is stored in the local database of each medical institution in an encrypted manner, and the summary information of the ERMR is stored on the consortium blockchain.

The detailed information of the ERMR includes the rehabilitation doctor ID, patient ID, ciphertext of the ERMR, keyword index, and digital signature of the rehabilitation doctor (see Figure 5). The ciphertext of the medical record is encrypted using the patient's public key, and its content mainly includes the encrypted description of the condition, examination records, treatment records, and consultation time. The keyword index extracts meaningful words from the original record of the ERMR as an index, pointing to the storage location of the ERMR file. The digital signature of the rehabilitation doctor is used to verify the identity of the doctor to ensure the authenticity of the rehabilitation medical data.

The summary information of ERMR is stored on the consortium blockchain using a blockchain data structure. The hospital server creates a new block at regular intervals, in which the summary information of ERMR is stored, and all the blocks are connected into a chain in the order of creation time. Each block consists of two parts: the block header and the block body (see Figure 6).

In the block header, the block hash is the hash value used to uniquely identify the block. The blocks are linked by the hash value of the previous block (that is, the parent hash). The block timestamp records the generation time of each block. In the block body, the ERMR summary information is stored in a Merkle tree structure, which can be used to verify the authenticity and integrity of medical data. The main content of the ERMR summary information includes hospital server ID, patient ID, keyword index, digital signature of the hospital server, and transaction timestamp. The digital signature of the hospital server is used for identity verification to ensure that the data on the blockchain is authentic and reliable. Transaction timestamp records the entry time of each summary information, accurate to the millisecond. It adds a time dimension to the rehabilitation medical data, making it easier to trace and supervise.

The ERMR do not need to be shared globally, only the super nodes on the consortium blockchain can obtain the summary information of ERMR. When medical institutions need to query external data, the consortium blockchain forwards the query request to the provider of the original ERMR based on the ERMR summary information. This method realizes the separation of block data and business data, so that medical institutions can not only realize the point-to-point query of ERMR, but also reduce the risk of medical data leakage. In addition, it can effectively reduce the pressure of high-frequency access to the consortium blockchain and ensure the read and write performance of the block data.

### 4.3. The Data Transmission Mode Design

Before logging in to the blockchain system, doctors, patients, and third-party institutions need to register, create unique digital identities, and generate their own key pair, in which the public key is externally exposed, and the private key is not. The data transmission process is as follows (see Figure 7).

1. The patient goes to the hospital for treatment, and the patient's public key information is contained in the medical card
2. The rehabilitation doctor enters the ERMR for the patient, encrypts the ERMR with the patient's public key, and generates a keyword index. The detailed information of the ERMR such as the patient ID, ERMR ciphertext, and keyword index is stored in the hospital's local database
3. The hospital server creates a new block at regular intervals to upload the ERMR summary information such as the hospital server ID, patient ID, and keyword index to the consortium blockchain. Other nodes on the consortium blockchain are responsible for verifying the transaction, and if the verification is passed, the new block is created
4. When the patient goes to other hospitals, if the rehabilitation doctor needs to know the patient's medical history, he can search through the ERMR summary information on the consortium blockchain and send the query request to the provider of the original ERMR. The data provider encrypts the detailed information of the ERMR with the patient's public key and sends it to the inquirer. After receiving the information, the inquiring party uses the patient's private key to decrypt the ERMR and read the content of the medical record with the patient's authorization. Without the authorization of the patient, the detailed information of the ERMR cannot be decrypted, thereby reducing the risk of the leakage of the patient's personal information and protecting the privacy and legal rights of the information subject
5. If a third-party institution (such as the insurance company, the rehabilitation research institution, etc.) needs to access the patient's ERMR, it needs to obtain the patient's authorization and decrypts the ERMR with the patient's private key. Smart contract can be used to achieve an automated incentive mechanism, and the more the patient's ERMR is queried, the greater the value of the data. The patients can get rewards from ERMR sharing, thereby ensuring the economic interests of the information subject and returning the data ownership to the patient

### 4.4. The Digital Signature Design

First, the private key *k* and the public key *K* of the sender's hospital server need to be generated. The description of the relevant variables is as follows.

*M*-plaintext of the ERMR.

*h*-hash value of the ERMR.

*G*(*x*, *y*)-base point on the elliptic curve.

*k*-private key of the sender.

*K*-public key of the sender.

*r*-random number.

Take a base point *G*(*x*, *y*) on the elliptic curve and set *K* = *kG*(*x*, *y*). The specific process for the hospital server to generate a digital signature is as follows (see Figure 8).

1. Use a hash function to map information *M* to a hash value *h*
2. Choose a random number *r* and calculate the point *rG*(*x*, *y*)
3. Use the private key *k* of the hospital server to encrypt the hash value *h*, calculate *s* = *h* + *kx*/*r*, and get the digital signature {*rG*(*x*, *y*), *s*}
4. Upload the information *M* and the digital signature {*rG*(*x*, *y*), *s*} to the consortium blockchain together

The specific process for the inquirer of the ERMR to verify the digital signature is as follows (see Figure 9).

1. Find the hash value *h* according to the information *M*
2. The receiver uses the public key *K* to decrypt the digital signature and calculate (*hG*(*x*, *y*)/*s*) + (*xK*/*s*)
3. Compare whether it is equal to *rG*(*x*, *y*), so as to verify whether the information comes from the sender

The derivation process of the verification principle is as follows.

(1) $$\begin{array}{c} \frac{\text{hG}\left(\text{x},\text{y}\right)}{\text{x}}+\frac{\text{xK}}{\text{s}}=\frac{\text{h}}{\text{s}}\text{G}\left(\text{x},\text{y}\right)+\frac{\text{x}}{\text{s}}\text{kG}\left(\text{x},\text{y}\right)=\frac{\text{h}+\text{kx}}{\text{s}}\text{G}\left(\text{x},\text{y}\right)=\frac{\text{r}\left(\text{h}+\text{kx}\right)}{\text{h}+\text{kx}}\text{G}\left(\text{x},\text{y}\right)=\text{rG}\left(\text{x},\text{y}\right). \end{array}$$

### 4.5. The Consensus Algorithm Design

ERMR sharing based on the consortium blockchain is an application scenario in a trusted environment, and the security is higher than the public blockchain scenario; so, the consensus algorithm is more suitable for the non-Byzantine Raft algorithm, which can achieve data consistency under the premise that more than half of the nodes in the system are operating normally. The Raft algorithm divides time into a series of terms. During each term, all nodes vote to elect a leader. The leader is given the right to keep accounts during the term and is responsible for generating the new blocks. Until the next term, the system elects a new leader.

Each node in the consortium blockchain has three states: leader, follower, and candidate. Under the normal circumstances, there is only one leader in one term, and all other nodes are followers. When the follower does not receive a response from the leader for a certain period of time (usually 150-300 milliseconds), the system converts to the candidate state, and a new leader needs to be elected.

Assuming there are *N* nodes in the consortium blockchain, *R*_1_, *R*_2_,…, *R*_*N*_ represent the nodes in the consortium blockchain, *S*_1_, *S*_2_,…, *S*_*N*_ represent the state of each node (i.e., leader, follower, or candidate), and *v* represents the number of affirmative votes. The leader election steps are as follows (see Algorithm 1).

1. In the candidate state, the node *R*_1_ sends a REQUEST to the other *N-*1 nodes, requesting to elect itself as the leader
2. If other nodes agree, then vote for it
3. When the affirmative votes reach (*N*/2) + 1, it means that the affirmative votes account for the majority, the node *R*_1_ becomes the leader, and the other nodes become the followers

After the leader *R*_1_ is selected, the process of log replication is as follows (see Algorithm 2), in which *u* represents the number of nodes who agree to append the record, and *c*_1_, *c*_2_*,…,c*_*N*_ represent the state of the new record (i.e., committed or uncommitted) in the node *R*_*i*_.

1. The client sends a REQUEST to append a new transaction record to the leader *R*_1_
2. The leader *R*_1_ appends the new record to its log
3. The leader *R*_1_ issues an INSTRUCTION to all the followers, asking them to append the new record to their respective logs
4. When most of the followers agree to append the record to their logs, the addition of the record is confirmed, and then the leader *R*_1_ will send the client a MESSAGE of successful record entry
5. The leader *R*_1_ informs all the followers to add the confirmed record to their logs

During this process, if a network communication failure occurs and the leader *R*_1_ cannot access most of the followers, the blockchain system will switch to the candidate state and the leader will be reelected. During the loss of connection, any update of the original leader *R*_1_ cannot be confirmed, and all transactions will be rolled back.

## 5. Results and Discussion

### 5.1. Results

The ERMR sharing scheme proposed in this paper can be developed and deployed on the basis of the Hyperledger Fabric framework, and smart contracts are written in Go language. In the smart contract, the Go program code to import the Fabric framework is as follows:

  import (“github.com/hyperledger/fabric/core/chaincode/shim”sc“github.com/hyperledger/fabric/protos/peer”)

Define a struct in the smart contract to store the ERMR summary information, and the code is as follows:

  type Summary struct {ServerId string PatientId string Keyword string
  }

In order to verify the feasibility of the scheme, 110 rehabilitation electronic medical records were collected as test cases. In the Fabric1.4 environment, five orderer nodes (i.e., orderer 1, orderer 2, orderer 3, ordererer 4, and orderer 5) were built to provide the consensus service. The configuration of the test environment is shown in Table 3.

First, stop the server of Orderer5, and the system can respond to the client request normally. Then, stop the server of Orderer4, and the system can still respond to the client request normally. Then, stop the server of Orderer3, and at this time, the client's request cannot be responded to. As can be seen, under the action of the Raft consensus algorithm, data consistency can be achieved, and the blockchain network with 5 nodes can tolerate the failure of up to 2 nodes.

### 5.2. Discussion

The scheme proposed in this paper helps to realize the safer and faster sharing of ERMR, the rehabilitation hospitals, rehabilitation centers, communities, insurance companies, research institutions, government departments, and other institutions can benefit from it, so as to better facilitate the development of smart healthcare. The scheme proposed in this paper has the following potential application scenarios.

Diagnosis and treatment of chronic diseases. Patients with chronic diseases need long-term and continuous treatments, and various related parties are involved during the treatment, such as rehabilitation doctors, rehabilitation therapists, and third-party service agencies. The ERMR sharing scheme based on blockchain technology can break the access barriers between different medical institutions, so that the doctors can track the patient's historical diagnosis and treatment and reduce the waste of resources caused by repeated diagnosis and treatment. It can establish trust between various stakeholders, so that all relevant parties can share information in a protected environment and realize the full-process sharing and collaboration of chronic disease treatment.

Supervision and control of rehabilitation medical services. The rehabilitation medical record is an important basis for handling medical disputes. However, under the current technical conditions, rehabilitation medical record may be tampered with when a medical accident occurs, which makes it difficult to provide evidence and determine responsibility, and cause escalation of doctor-patient conflicts. The nontamperable feature of blockchain can solve this problem. In the event of a medical accident, the specific responsible person can be identified, achieving the effective control of the quality of rehabilitation medical services.

Medical insurance claims. The current process of medical insurance claims usually involves the applicant paying the treatment fee to the hospital first and then claiming compensation from the insurance company after obtaining the payment list from the hospital. The whole process is complicated and time-consuming. By using the blockchain technology, the insurance company can obtain the medical expense data in real time. Smart contract can realize the automatic verification of insurance contracts and automatic execution of claims, thereby improving the efficiency of claims processing. The nontamperable feature of blockchain can effectively reduce the medical fraud caused by tampering with medical records.

Clinical research in rehabilitation medicine. ERMR sharing can provide important basic data and case reports for clinical research of rehabilitation medicine. On this basis, rehabilitation researchers can perform medical record analysis and data mining to better serve the rehabilitation clinical treatment.

Supervision and traceability of rehabilitation medicine. Regulatory authorities can obtain credible rehabilitation medical data in real time, grasp the overall status of residents' chronic diseases, and evaluate the overall living conditions of disabled people in society, thus greatly improving the efficiency of supervision and providing a basis for formulating relevant policies.

## 6. Conclusions

Specifically, the contributions of this paper mainly included the following aspects.

This paper adopted a hybrid P2P network structure, used hospitals, research institutes, insurance companies, civil affairs departments, and other institutions as super nodes, designed a hybrid P2P structure alliance chain. While realizing the distributed storage of ERMR, the controllability of the system was better maintained.

An on-chain-off-chain hybrid storage mechanism was designed in this paper. The detailed information of the ERMR was stored in the local database of each hospital, and the summary information of the ERMR was stored on the consortium blockchain in a block-chain data structure. This storage mechanism could not only realize the point-to-point query of ERMR between different hospitals but also effectively solve the attack problem under the centralized storage on third-party cloud servers, thereby effectively reducing the risk of medical data leakage and ensuring the read and write performance of data on the blockchain under the condition of increasing data volume.

The asymmetric encryption algorithm was used in this paper to realize the safe sharing of ERMR. The public key and private key were used to encrypt and decrypt the ERMR. The private key was not transmitted on the blockchain network, which greatly reduced the risk of information leakage. Only after being authorized by the patient and obtaining the patient's private ke, could the medical institution be able to read the content of the ERMR, thereby strengthening the protection of the patient's personal information and avoiding the legal and ethical risks caused by medical data sharing in the traditional way.

The digital signature technology was used to realize the identity verification of the hospital server and strengthen data security. Based on the hash algorithm and asymmetric encryption algorithm, the digital signature has been designed. When the hospital server sent the information, it encrypted the hash value of the information with its own private key as a signature and sent the information and the signature to the receiver. The receiver used the message, signature, and the sender's public key to perform calculation and comparison. If they were consistent, the verification passed.

Based on the Raft algorithm, the consensus mechanism of the consortium blockchain was designed, which could solve the system crash caused by node server failure or network communication failure, thereby effectively improving the fault tolerance of the system and ensuring the consistency of data in the blockchain network.

## Figures and Tables

**Figure 1:** The P2P network structure.

**Figure 2:** The blockchain data structure.

**Figure 3:** The basic principle of asymmetric encryption algorithm.

**Figure 4:** The hybrid P2P network structure.

**Figure 5:** The storage structure of the detailed information of ERMR.

**Figure 6:** The storage structure of the ERMR summary information.

**Figure 7:** The transmission process of the rehabilitation data.

**Figure 8:** The generation process of digital signature.

**Figure 9:** The decryption process of digital signature.

**Algorithm 1:** Algorithm on leader election

**Algorithm 2:** Algorithm on log replication

**Table 1:** Main data content of rehabilitation medical record.

Data category	Main content
Patient identification	Name, ID number, gender, date of birth, home address, etc.
General health	Nutritional status, excretion method, bowel function, sleep mode, safety issues, mental status, language, hearing, vision, activity status, self-care status, etc.
Past medical history	History of disease, infectious disease, allergy, vaccination, surgery, trauma, blood transfusion, etc.
History of present illness	The cause, main symptoms, duration, degree of impact of the dysfunction, the status of receiving rehabilitation treatment, etc.
Professional and psychosocial history	Occupation, lifestyle, economic status, history of marriage and childbirth, family status, living environment, mental state, interests and hobbies, etc.
Physical examination	Body temperature, pulse, blood pressure, respiration, weight, urinalysis, skin damage, etc.
Specialist examination	Nervous system and musculoskeletal system examination and measurement, such as advanced brain function, neural reflex, gait analysis, joint range of motion, muscle tone, hand muscle strength, balance disorder, and upper and lower limb function
Functional rating scale	Activity of Daily Living Scale (ADL), NIH Stroke Scale (NIHSS), European Stroke Scale (ESS), Brunnstorm Motor Function Rating, Fugl-Meyer Assessment (FMA), wolf motor function test (WMFT), manual muscle testing (MMT), range of motion (ROM), Modified Rankin Scale (MRS), Modified Ashworth Scale (MAS), Berg Balance Test, Function Independent Measure (FIM), Modified Barthel Index (MBI), etc.
Laboratory and instrument examination	Center of gravity measurement, stability limit evaluation, smart Equitest balance master, imaging examination, etc.
Diagnosis	Disease diagnosis, dysfunction diagnosis, complications, etc.
Treatment plan	Preliminary rehabilitation goal, rehabilitation method (such as physical therapy, occupational therapy, speech therapy, etc.), types of medications, prevention of systemic risks in rehabilitation medicine, etc.
Rehabilitation assessment	Short-term and long-term goals of rehabilitation treatment, current treatment plan, treatment points, and precautions

**Table 2:** The smart contracts of mainstream blockchain platforms.

Blockchain platform	Development language	Operating environment
Bitcoin	Script	/
Ethereum (ETH)	Solidity/serpent	EVM
Hyperledger Fabric	Go/Java	Docker
R3 Corda	Kotlin/Java	JVM

**Table 3:** Configuration of the test environment.

Item	Version/parameter
Operating system	Ubuntu 16.04 TLS
CPU	Intel i7 7700
Memory	16G DDR4
Hard disk	1 T HDD
Hyperledger Fabric	1.4.1

## Data Availability

The electronic rehabilitation medical record data used to support the findings of this study are included within the article.
